# Semisupervised Seizure Prediction in Scalp EEG Using Consistency Regularization

**DOI:** 10.1155/2022/1573076

**Published:** 2022-01-25

**Authors:** Deng Liang, Aiping Liu, Le Wu, Chang Li, Ruobing Qian, Rabab K. Ward, Xun Chen

**Affiliations:** ^1^The Epilepsy Center, Department of Neurosurgery, The First Affiliated Hospital of USTC, Division of Life Sciences and Medicine, University of Science and Technology of China, Hefei 230001, China; ^2^School of Information Science and Technology, University of Science and Technology of China, Hefei 230027, China; ^3^Department of Biomedical Engineering, Hefei University of Technology, Hefei 230009, China; ^4^Department of Electrical and Computer Engineering, University of British Columbia, Vancouver, British Columbia V6T 1Z4, Canada

## Abstract

Early prediction of epilepsy seizures can warn the patients to take precautions and improve their lives significantly. In recent years, deep learning has become increasingly predominant in seizure prediction. However, existing deep learning-based approaches in this field require a great deal of labeled data to guarantee performance. At the same time, labeling EEG signals does require the expertise of an experienced pathologist and is incredibly time-consuming. To address this issue, we propose a novel Consistency-based Semisupervised Seizure Prediction Model (CSSPM), where only a fraction of training data is labeled. Our method is based on the principle of consistency regularization, which underlines that a robust model should maintain consistent results for the same input under extra perturbations. Specifically, by using stochastic augmentation and dropout, we consider the entire neural network as a stochastic model and apply a consistency constraint to penalize the difference between the current prediction and previous predictions. In this way, unlabeled data could be fully utilized to improve the decision boundary and enhance prediction performance. Compared with existing studies requiring all training data to be labeled, the proposed method only needs a small portion of data to be labeled while still achieving satisfactory results. Our method provides a promising solution to alleviate the labeling cost for real-world applications.

## 1. Introduction

Epilepsy is a chronic neurological disorder and affects around 50 million people worldwide [1]. It is characterized by recurrent seizures, which are abnormal involuntary movements of the entire or partial body and sometimes accompanied by unconsciousness. Up to 70% of the epileptic patients could live seizure-free with appropriate use of antiseizure medicines, while the other 30% are intractable. The drug-resistant patients have to endure recurrent unforeseeable seizures, which threaten their lives and limit daily activities [2]. In such a case, a precise prediction of the upcoming seizure would be of great value as it allows the patients to adjust behaviors and take precautions against possible injuries.

Electroencephalography (EEG) is a powerful and convenient tool in the recording and measuring of bioelectrical brain activity [3, 4], being able to detect brain abnormalities precisely. Over the last few years, studies have shown that epileptic seizures can be predicted by EEG [5, 6]. Most studies divided the consecutive epileptic EEG signals into four states: preictal (a short period before a seizure), ictal (during the seizure), postictal (the period after a seizure), and interictal (the period between seizures other than preictal and postictal). In general, epileptic seizure prediction can be described as a binary classification problem that distinguishes between the preictal and interictal. Specifically, an alarm will be raised if the state is detected as preictal, warning the patient to take precautions. In the literature, most methods aim to improve prediction accuracy.

Traditional methods primarily consist of three procedures, including preprocessing (e.g., denoising and normalization), feature extraction, and classification [6]. Among these steps, feature extraction is the most crucial step, aiming to derive a discriminative biomarker from physiological signals. In previous studies, the extracted features could be categorized into two main groups: linear and nonlinear features. Spike rate [7], spectral band power [8], spectral edge frequency, and Hjorth parameters [9] have been introduced as linear features. On the other hand, several nonlinear features, derived from the theory of dynamic systems, have been developed, such as dynamic similarity index [10], Lyapunov exponent [11], and phase synchronization [12]. After feature extraction, a variety of classifiers are carried out to make identification decisions, like random forest [13] and support vector machine (SVM) [14]. Although the reported performances are very impressive, traditional methods rely on professional knowledge to construct reasonable hand-crafted features, and the constructed features may not be optimal all the time due to the dynamic changes of the brain [15].

In recent years, deep learning has been introduced into this field with great success due to its strong automatic feature extraction ability. Khan et al. applied convolutional neural network (CNN) to identify preictal and interictal phases, using the wavelet transformation (WT) of the EEG signals as input [16]. Truong et al. presented a seizure prediction model exploiting the short-time Fourier transformer (STFT) time-frequency representation as the input of CNN [15]. Ahmet and Sarp used spectral band power, statistical moment, and Hjorth parameters to construct 3D representations according to the topology of the EEG channels and applied 3D CNN to perform seizure prediction [17]. Zhang et al. proposed employing common spatial pattern (CSP) as the input of CNN for seizure prediction [18]. Wang et al. employed directed transfer function (DFT) to explore the specific information exchange between EEG channels and then used CNN for seizure prediction, achieving satisfactory performance [19].

However, the success of deep learning approaches highly relies on the abundance of labeled training data. In practice, labeling EEG signals does require the expertise of an experienced pathologist and is incredibly time-consuming [20]. On the contrary, unlabeled data are easy to obtain but hard to utilize for training. It is of great value if we can take advantage of extensive unlabeled data rather than limited manually annotated data [21]. To solve this problem, in this paper, we introduce semisupervised learning which can make use of both labeled and unlabeled data. Numerous semisupervised deep learning methods have been proposed in various fields [22, 23]. Inspired by the success of consistency regularization in image classification [24], we present a novel solution called Consistency-based Semisupervised Seizure Prediction Model (CSSPM), where only a small portion of training data is labeled. Consistency regularization underlines that a robust model should maintain consistent results for the same input under extra perturbation. It provides a way to learn about the underlying structure of the data from unlabeled samples and produces a better estimate of the decision boundary. A schematic illustration of the consistency regularization is given in Figure 1. When trained only on the limited labeled data in a supervised manner, the neural network is easy to overfit, and the decision boundary does not follow the “manifold” of the data. On the other hand, in a consistency regularization-based method, appropriate perturbations are added to an input sample *x* to generate an augmented sample *x*′ and a regularization loss is applied to minimize the difference between the predictions *f*(*x*) and *f*(*x*′). This operation does not require a label and is known to make the decision boundary far away from the high-density region [25].

In our study, we adopt Gaussian noise and dropout as perturbations so that the entire neural network could be regarded as a stochastic model. During training, the same input would yield different results at different epochs. Then we construct a consistency constraint to penalize the difference between the current prediction and previous predictions. To better verify the effectiveness of our proposed semisupervised strategy, the network architecture, as well as the parameters, completely follows the work in [15]. Compared with the baseline, where all training data are labeled, our method only needs a small portion of training data to be labeled with the rest training data unlabeled.

The main contributions of this paper are concluded as follows:

1. We present a novel semisupervised framework called Consistency-based Semisupervised Seizure Prediction Model (CSSPM) to alleviate the labeling cost. The CSSPM is able to learn information from unlabeled data. Specifically, by using stochastic augmentation and dropout, we consider the entire neural network as a stochastic model and design a consistency regularization to penalize the difference between the current prediction and previous predictions. This operation is able to improve the decision boundary without label information.
2. We design a joint training objective driving the model to learn information from both labeled and unlabeled seizure data simultaneously. To the best of our knowledge, this is the first study to perform seizure prediction with a small portion of labeled seizure data.

## 2. Materials and Methodology

### 2.1. Dataset

In this study, the CHB-MIT scalp EEG database, collected at the Children's Hospital Boston, is used to train and test the model [26, 27]. The dataset contains 23 long-duration recordings from 22 patients with intractable epilepsy. Most cases included 23 channels according to the 10–20 international system, and all these multichannel EEG signals were acquired with a 256 Hz sampling rate.

Following [15], we introduce the definition of some relevant parameters. The preictal period is defined as 30 minutes before the onset of a seizure, while the interictal period is defined as more than four hours before the onset of a seizure and more than four hours after the end of a seizure. In the case of two seizures occurring at a short interval, the latter seizure is not evaluated, and the preictal period of the leading seizure is only left. The minimum interval is set to 30 minutes. Besides, it is not that critical to perform seizure prediction for patients who suffer seizures too frequently; therefore, only patients who suffered seizures less than ten times per day are considered. To ensure that there are enough unlabeled data in the training set (clarified in subsection 2.3.2), we choose patients who had at least four leading seizures while the baseline only requires patients having at least three seizures. With these definitions, we select 11 patients for our experiments and summarize the subject information in Table 1.

### 2.2. Preprocessing

We follow the same preprocessing steps with [15]. The consecutive recordings are divided into 30-second EEG segments and then converted into image shape by the short-time Fourier transform (STFT). To remove the power line noise at 60 Hz, we exclude the components in the frequency ranges of 57–63 Hz and 117–123 Hz. And the DC component (at 0 Hz) is also excluded. For the data imbalance problem, where the preictal data are much less than the interictal, we generate more preictal samples in training set by an overlapped sampling technique. Specifically, we slide the 30-s window along the time-axis at a step of *S*, where *S* is calculated per patient to make the number of preictal samples close to interictal samples.

### 2.3. Consistency-Based Semisupervised Seizure Prediction Model

In this subsection, we clarify how we train the model using a small portion of labeled data as well as an amount of unlabeled data. The overall structure of CSSPM is described in Figure 2, and the pseudocode is shown in Algorithm 1. We take the STFT as input and utilize CNN to learn the feature, where the parameters are set as same as [15]. The training set includes both labeled and unlabeled samples. The labeled samples are evaluated using standard cross-entropy loss. In addition, a consistency loss is applied to both the labeled and unlabeled samples.

#### 2.3.1. Network with Dropout

As shown in Figure 3, the architecture is lightweight, including three convolution blocks. In each block, a batch normalization layer, a convolution layer with ReLU activation, and a max-pooling layer are built in turn. The first block uses 3D convolution to filter the STFT representations having 16*n* × 5 × 5 kernels with a stride of 1 × 2 × 2, where *n* is equal to the number of input channels. A 1 × 2 × 2 max-pooling layer is applied for downsampling. Then the output feature maps are reshaped into the 2D format and exploited by the subsequent two blocks. The following two blocks adopt 2D convolution with 32 and 64 kernels, respectively, and both use 3 × 3 kernels with a stride of 1 × 1 and 2 × 2 max-pooling. Finally, the features of these convolution blocks are flattened and further explored by two fully connected layers to generate the final prediction of the input segments. The first fully connected layer has 256 units with a sigmoid activation, while the second fully connected layer has two units with a softmax activation. Both of them have a dropout rate of 0.5.

#### 2.3.2. Training and Testing Strategy

Let *D* represent the whole training set, and *L* represent the index set of the labeled data. The STFT input is denoted *x*_*i*_, where *x*_*i*_ ∈ *D*. Only for the labeled data *i* ∈ *L*, the ground truth is given, *y*_*i*_ ∈ {0,1}, where 0 denotes the interictal sample, and 1 denotes the preictal sample. During training, for each input sample *x*_*i*_ , the model generates the prediction vectors *z*_*i*_ :

(1) $$\begin{array}{c} z_{i}=f_{\theta }\left(g\left(x_{i}\right)\right),\;x_{i}\in D, \end{array}$$

where *f*_*θ*_ denotes the network with trainable parameters *θ* and *g* means the Gaussian augmentation function.

After every epoch, we construct ensemble prediction by integrating the current prediction and previous predictions:

(2) $$\begin{array}{c} Z_{i}=\alpha Z_{i}+\left(1-\alpha \right)z_{i}, \end{array}$$

where *Z*_*i*_ denotes the ensemble prediction using a moving weighted average from the previous predictions to the current prediction and *α* is the ensemble constant. To correct the startup bias, we divide the ensemble prediction by factor (1 − *α*^*t*^), generating the final target $\tilde{Z_{i}}$:

(3) $$\begin{array}{c} \tilde{Z_{i}}=\frac{Z_{i}}{1-\alpha^{t}}. \end{array}$$

It is worth mentioning that, under the Gaussian noise augmentation and dropout regularization, the output prediction is regarded as a stochastic variable. And there would always be a bias between the prediction *z*_*i*_ and $\tilde{Z_{i}}$, which can be regarded as an error in classification. Therefore minimizing this bias is reasonable and makes the model more stable.

In this study, the loss function of CSSPM consists of two components. The first component takes the supervised cross-entropy loss to evaluate labeled data only, enforcing the prediction consistent with the ground truth. The second component takes the unsupervised mean square error loss to penalize the bias between different predictions for the same input, evaluated for all training data. What is noteworthy is that the perturbations cause minor variations in the input space but are not enough to change the properties of the EEG signal. The augmented inputs from different epochs are highly similar and, more critically, always belong to the same category. While the consistency constraint requires minor variations in the output space, it implies to the model that similar inputs should belong to the same class so that the decision boundary will be pushed far away from the high-density region [28].

The cross-entropy loss evaluated for labeled data is defined as follows:

(4) $$\begin{array}{c} L_{c}=-\frac{1}{\left|B\right|}\sum_{i\in \left(B\cap L\right)}-y_{i}\log\left(z_{i}\right)-\left(1-y_{i}\right)\log\left(1-z_{i}\right), \end{array}$$

where *B* means the current minibatch, and the unsupervised mean square error loss is given as follows:

(5) $$\begin{array}{c} L_{con}=\frac{1}{C|B|}\sum_{i\in B}{\left\|z_{i}-\tilde{Z_{i}}\right\|}^{2}, \end{array}$$

where *C* denotes the number of categories. As the confidence of the prediction of unlabeled data is often deficient in the beginning, when combining the supervised component and the unsupervised component, we weight the latter by a ramp-up weighting function *ω*(*t*). The weight increases gradually from 0 to the maximum, and the supervised component dominates the learning of the network at early epochs.

(6) $$\begin{array}{c} L=L_{c}+\omega \left(t\right)L_{con}. \end{array}$$

The ramp-up weighting function *ω*(*t*) is defined as

(7) $$\begin{array}{c} \omega \left(t\right)=\left\{\begin{array}{cc} \exp\left[-5{\left(1-\frac{t}{\tau }\right)}^{2}\right]*\omega_{\max}, & t⩽\tau ,\\ \omega_{\max}, & t>\tau . \end{array}\right. \end{array}$$

The prediction algorithm is evaluated in a patient-specific manner using leave-one-out cross-validation [15]. To be specific, if a patient has *N* defined seizures, there are *N* corresponding preictal periods. We firstly divide the interictal data into *N* parts and combine them with preictal data to generate “*N* seizure recordings.” In these *N* recordings, each recording is left aside as the testing data in turn, and the remaining (*N* − 1) recordings are used for training and validation. For these *N* − 1 recordings, one recording is randomly selected as the validation set, and the rest are used as the training set. In the training set, we randomly select one recording as the labeled set while the other multiple recordings are left unlabeled. In brief, as illustrated in Figure 4, we take one labeled seizure recording and (*N* − 3) unlabeled seizure recordings for training and take another labeled recording as the validation set. To ensure the existence of unlabeled data, we choose patients with at least four seizures (*N* − 3 > 0). During training, the accuracy of the validation set is calculated to determine whether the model is overfitting the training set. The training would be terminated when the accuracy of the validation set has reached the maximum, and the model at the corresponding moment is adopted for testing. The process repeats *N* times until every seizure recording has been tested and an averaging result is calculated.

### 2.4. Postprocessing

The network output only expresses the state of a 30-s segment, and we need to synthesize multiple predictions to determine whether to trigger an alarm. We adopt the *k*-of-*n* method, where an alarm is triggered only if at least *k* outputs during the last *n* outputs were detected to be preictal [15]. The parameters are set to *k*=8 and *n*=10. This means if during the last 300 s the system reports preictal more than 240 s, the alarm will be triggered. Besides, to prevent continuous alarms from occurring for a short time, we set the refractory period to 30 mins.

## 3. Experiments and Results

To verify the effectiveness of CSSPM, we conduct extensive experiments on the CHB-MIT scalp EEG database. In this section, we will introduce the evaluation metrics, the experiment settings, and the results.

### 3.1. Evaluation Metrics

Before estimating the performance, we need to define the seizure occurrence period (SOP) and the seizure prediction horizon (SPH) in advance. The SOP is the period in which seizures are predicted to occur, while the SPH is the period between seizure alarm and the onset of the SOP [29]. The SPH is also called intervention time, allowing patients to take precautions. The prediction is correct only when the seizure occurs within the SOP; otherwise, it is judged as a false alarm. The illustration is given in Figure 5. In our experiments, the SPH is set to 5 minutes, and the SOP is considered 30 minutes.

Two main metrics, the sensitivity, and the false alarm prediction rate (FPR) are used to evaluate the performance [15]. The sensitivity is defined as the proportion of seizures that are correctly predicted, while the FPR indicates the number of false alarms per hour. Specifically, the exact formulas of sensitivity are expressed as follows:

(8) $$\begin{array}{c} \text{sensitivity}=\frac{TP}{FN+TP}\times 100\%, \end{array}$$

where TP denotes the number of seizures that are correctly predicted, and FN represents the number of seizures that are missed. The FPR is given in

(9) $$\begin{array}{c} FPR=\frac{FP}{\text{time}\left(\text{interictal}\right)}. \end{array}$$

where FP denotes the number of false alarms.

In addition, we calculate *p* values according to [30], which is used to compare the method with a random predictor. The probability of raising an alarm by the random predictor with the same FPR can be approximated by

(10) $$\begin{array}{c} prob\approx 1-e^{-FPR\cdot SOP}. \end{array}$$

Then the probability of predicting at least *k* of *K* seizure events by this predictor can be calculated by

(11) $$\begin{array}{c} p=\sum_{i\geq k}\left(\begin{array}{c} K\\ i \end{array}\right)prob^{i}{\left(1-prob\right)}^{K-i}. \end{array}$$

The *p* value is calculated for every patient using the same FPR and the number of correctly predicted seizures (*k*) obtained by our method. When *p* < 0.05, it is concluded that the algorithm achieves significantly better results than a random predictor.

### 3.2. Experiment Settings

In this subsection, we introduce the experiment settings. The standard deviation of the additive Gaussian noise is set to *σ*=0.15. The model is trained using Adam optimizer with a maximum learning rate of *λ*_max_=0.0005, and the momentum parameters are set to *β*_1_=0.9 and *β*_2_=0.999. The minibatch size is set to |*B*|=32, and the maximum number of epochs is set to 50. For the ramp-up weighting function *ω*(*t*), the parameters are set to *ω*_max_=30 and *τ*=30. Similar to the ramp-up *ω*(*t*), we adopt the Gaussian curve to ramp down the learning rate, but time-reversed and the scaling constant is set to 12.5 instead of 5. The ensembling constant is set to *α*=0.6 in all runs. We do the experiments using Python libraries and Keras 2.1.6 framework on a server with Xeon E5 2620 CPU and four NVIDIA 2080Ti graphics cards.

### 3.3. Results

In our study, we train the model using only one labeled seizure recording and multiple unlabeled seizure recordings. To verify the effectiveness of our proposed semisupervised strategy, we compare our model with the baseline that only uses standard cross-entropy. When training the baseline on only one labeled seizure recording, the labeled recording and validation set are exactly the same as CSSPM. In the leave-one-out cross-validation, each fold is executed twice, and the average results with standard deviations are reported [15]. Since we completely follow the data processing in the original baseline and the testing set is totally the same, we use their results reported in the literature directly to make a fair comparison.

Table 2 shows the prediction results of the baseline and CSSPM. The original baseline using all labeled data, the baseline trained on only one labeled recording, and CSSPM achieve an average sensitivity of 82.6%, 62.9%, and 78.5%, respectively, for the selected patients. Accordingly, the FPR is calculated as 0.21 h, 0.70 h, and 0.44 h. The significant level p is set to 0.05, and the number of patients in which the algorithm works significantly better than a chance predictor (*p* < 0.05) is 10, 6, and 8, respectively. Comparing these results, when the amount of labeled data decreases sharply, the performance of the baseline declines obviously, because the model is more likely to overfit and performs poorly on the testing data. By fully exploiting the unlabeled data, the performance of CSSPM is significantly better than the baseline trained on the same labeled recording and very close to the original baseline.

We further compare these methods while increasing the proportion of labeled data in the training set. The number of labeled recordings increases gradually from 1 to 3. As stated in subsection 2.3.2, if a patient has *N* seizures, there is one labeled seizure recording for testing, one labeled seizure recording for validation, *n* labeled seizure recordings, and (*N* − 2 − *n*) unlabeled seizure recordings for training. To ensure the existence of unlabeled data, we have to choose patients who had enough seizure events (*N* − 2 − *n* > 0). Hence, as the number *n* increases gradually from 1 to 3, we choose four patients who had at least six seizure events, namely Pat1, Pat3, Pat10, and Pat18. The results are summarized in Table 3. With the increase of the proportion of labeled data, the performance of the baseline and CSSPM both improve gradually. In all experiments, CSSPM achieves superior results than the baseline. When three recordings are labeled in the training set, compared with the original baseline using all labeled data, CSSPM obtains almost the same average sensitivity with a little higher FPR value.

## 4. Discussion

Semisupervised learning is conceptually situated between supervised learning and unsupervised learning. A semisupervised algorithm always consists of a supervised component requiring labeled data and an unsupervised component using unlabeled data. Some semisupervised algorithms have been proposed in seizure prediction. Truong et al. presented a semisupervised method using a Generative Adversarial Network (GAN) [31]. The GAN was trained in an unsupervised manner, and then the extracted features from the trained discriminator were used for the seizure prediction task directly. This study proved that deep learning-based feature extraction could be performed in an unsupervised manner. Daoud et al. presented an autoencoder-based semisupervised model [32]. After the unsupervised reconstruction task, the pretrained encoder was adopted for the seizure prediction task directly, which could enhance the model optimization and help the model converge faster. Nasseri et al. proposed a semisupervised technique for seizure prediction in canines [33]. As the data are large in volume, they used unsupervised hierarchical clustering to select the preictal data most distinguishable from the interictal for classification and improve the performance effectively. Among these methods, unsupervised learning is exploited as the first step and then provides assistance to the following supervised learning. Therefore, they still require an amount of labeled data in the classification stage and have not alleviated the labeling cost. In our study, we make full use of unlabeled data to improve the decision boundary directly in classification and reduce the reliance on label information. To the best of our knowledge, this is the first study to perform seizure prediction with only a fraction of labeled data.

As consistency regularization is applied to all of the data, a concern exists that consistency regularization works mainly on labeled data, while unlabeled data are irrelevant. Considering this situation, we design an ablation experiment where unlabeled data are removed.  Table 4 shows that the performance of CSSPM without unlabeled data decreases obviously, and it demonstrates the effectiveness of unlabeled data.

In this study, we use Gaussian noise to add additional perturbation and force the network to resist its influence during training.  Table 5 presents the comparison between CSSPM with and without Gaussian augmentation. CSSPM with Gaussian augmentation obtains a sensitivity of 78.5% and a FPR value of 0.44 h. In contrast, CSSPM without Gaussian augmentation gets a sensitivity of 75.4% and a FPR value of 0.49 h. The introduction of Gaussian augmentation results in higher sensitivity and a lower FPR value, since training against additional perturbation can help the model to improve the decision boundary and increase robustness [28].

Finally, we discuss the limitation of this study and future works. Though the obtained sensitivity is close to the original baseline, the FPR value is still comparatively high, which means there is room for further improvement. As the presence of perturbation has a significant influence on the performance of semisupervised learning, except for the simple Gaussian noise, more stochastic augmentation strategies could be explored according to the characteristics of EEG. In this study, we build the convolutional neural network in keeping with [15], and different network architectures such as recurrent neural networks (RNN) and graph neural networks (GNN) might improve the performance, which is left for the future. In addition, we will extend this approach to other seizure-related fields, such as seizure detection and seizure type classification.

## 5. Conclusion

In this study, we propose a novel consistency-based semisupervised seizure prediction model, where only one recording of the training set is labeled. Using stochastic augmentation and dropout, we consider the entire neural network as a stochastic model and apply a consistency constraint to penalize the difference between the current prediction and previous predictions. In this way, unlabeled data can be fully exploited to improve the decision boundary that better reflects the underlying structure of the data. The method is evaluated on the CHB-MIT scalp EEG database using leave-one-out cross-validation. The results show that this semisupervised method achieves significantly better performance than the baseline under the same label information and performs even close to the original baseline with all labeled data. This study provides a promising solution to reduce the reliance on the label data in seizure prediction.

## Figures and Tables

**Figure 1:** A schematic illustration of the consistency regularization. When trained only on the limited labeled data in a supervised manner, the decision boundary does not follow the “manifold” of the data. On the other hand, consistency regularization could leverage unlabeled data to draw a decision boundary that better reflects the underlying structure of the data.

**Figure 2:** The overall structure of CSSPM. The loss function consists of two components. The first cross-entropy loss is evaluated for labeled inputs only, where the ground truth *y*_*i*_ is only given for these data. With the stochastic augmentation and dropout in the network, the entire neural network is considered as a stochastic model. The same input would yield different results at different epochs. Hence a mean square error loss, evaluated for all training data, is applied to penalize the bias between the current prediction *z*_*i*_ and the ensemble prediction $\tilde{Z_{i}}$. A ramp-up weighting function *ω*(*t*) is added to control the weight of the unsupervised mean square error loss.

**Figure 3:** The network architecture used in this study. It includes three convolution blocks, and in each block, a batch normalization layer, a convolution layer with ReLU activation, and a max-pooling layer are built in turn. The first block uses 3D convolution, while the next two adopt 2D convolution. The features of these convolution blocks are flattened and explored by two fully connected layers to generate the final prediction. Both of them have a dropout rate of 0.5.

**Figure 4:** The partitioning strategy for the seizure data. Assume that there are five seizure events.

**Figure 5:** Definition of the SOP and SPH. The prediction is correct only when the seizure occurs within the SOP.

**Algorithm 1:** The pseudocode of CSSPM.

**Table 1:** Data information of the selected patients in the CHB-MIT Scalp EEG Database.

Pat1	F	11	Frontal	7	17.0
Pat3	F	14	Frontal	6	21.9
Pat5	F	7	Frontal	5	13.0
Pat9	F	10	Temporal/occipital	4	12.3
Pat10	M	3	Temporal	6	11.1
Pat13	F	3	Temporal/occipital	5	14.0
Pat14	F	9	Frontal/temporal	5	5.0
Pat18	F	18	Frontal	6	23.0
Pat20	F	6	Temporal/parietal	5	20.0
Pat21	F	13	Temporal/parietal	4	20.9
Pat23	F	6	Temporal	5	3.0

**Table 2:** Seizure prediction performance achieved by the baseline and CSSPM for all 11 patients.

Patient	Baseline (trained on all labeled recordings)			Baseline (trained on one labeled recording)			CSSPM		
	Sensitivity (%)	FPR (h)	*p* value	Sensitivity (%)	FPR (h)	*p* value	Sensitivity (%)	FPR (h)	*p* value
Pat1	85.7 ± 0.0	0.24 ± 0.00	<0.001	85.7 ± 0.0	0.77 ± 0.06	0.005	100.0 ± 0.0	0.50 ± 0.03	<0.001
Pat3	100.0 ± 0.0	0.18 ± 0.00	<0.001	41.7 ± 8.3	0.16 ± 0.02	0.008	66.7 ± 0.0	0.12 ± 0.07	<0.001
Pat5	80.0 ± 20.0	0.19 ± 0.03	0.001	40.0 ± 0.0	0.35 ± 0.04	0.185	60.0 ± 0.0	0.46 ± 0.00	0.062
Pat9	50.0 ± 0.0	0.12 ± 0.12	0.067	50.0 ± 0.0	1.01 ± 0.20	0.519	50.0 ± 0.0	0.90 ± 0.08	0.459
Pat10	33.3 ± 0.0	0.00 ± 0.00	0.025	33.3 ± 0.0	1.26 ± 0.27	0.857	33.3 ± 0.0	0.45 ± 0.05	0.348
Pat13	80.0 ± 0.0	0.14 ± 0.00	<0.001	80.0 ± 0.0	0.18 ± 0.04	<0.001	90.0 ± 10.0	0.18 ± 0.05	<0.001
Pat14	80.0 ± 0.0	0.40 ± 0.00	0.004	60.0 ± 0.0	1.40 ± 0.00	0.506	80.0 ± 0.0	0.70 ± 0.10	0.029
Pat18	100.0 ± 0.0	0.28 ± 0.02	<0.001	50.0 ± 0.0	0.28 ± 0.02	0.033	83.3 ± 0.0	0.15 ± 0.02	<0.001
Pat20	100.0 ± 0.0	0.25 ± 0.05	<0.001	80.0 ± 0.0	0.15 ± 0.10	<0.001	100.0 ± 0.0	0.15 ± 0.00	<0.001
Pat21	100.0 ± 0.0	0.23 ± 0.09	<0.001	75.0 ± 0.0	0.55 ± 0.17	0.046	100.0 ± 0.0	0.41 ± 0.02	0.001
Pat23	100.0 ± 0.0	0.33 ± 0.00	<0.001	80.0 ± 0.0	1.50 ± 0.17	0.224	100.0 ± 0.0	0.83 ± 0.17	0.005
Ave	82.6 ± 1.8	0.21 ± 0.02	n.a	61.4 ± 0.8	0.70 ± 0.08	n.a	78.5 ± 0.9	0.44 ± 0.04	n.a

**Table 3:** Comparison of the baseline and CSSPM while increasing the number of labeled recordings in the training set (sensitivity/FPR).

Patient	Baseline (all labeled)	With one recording labeled		With two recording labeled		With three recordings labeled	
		Baseline	CSSPM	Baseline	CSSPM	Baseline	CSSPM
Pat1	85.7/0.24	85.7/0.77	100.0/0.50	85.7/0.38	100.0/0.44	85.7/0.16	100.0/0.15
Pat3	100.0/0.18	41.7/0.16	66.7/0.12	66.7/0.14	66.7/0.05	75.0/0.14	75.0/0.07
Pat10	33.3/0.00	33.3/1.26	33.3/0.45	41.7/0.72	50.0/0.50	58.4/0.72	58.4/0.68
Pat18	100.0/0.28	50.0/0.28	83.3/0.15	83.3/0.20	83.3/0.11	83.3/0.13	83.3/0.09
Ave	79.8/0.18	52.7/0.62	70.8/0.31	69.4/0.36	75.0/0.28	75.6/0.29	79.2/0.25

**Table 4:** The performance of CSSPM with and without unlabeled data.

Patient	Only labeled data			Labeled and unlabeled data		
	Sensitivity (%)	FPR (h)	*p* value	Sensitivity (%)	FPR (h)	*p* value
Pat1	100.0 ± 0.0	0.56 ± 0.03	<0.001	100.0 ± 0.0	0.50 ± 0.03	<0.001
Pat3	41.7 ± 8.3	0.18 ± 0.05	0.010	66.7 ± 0.0	0.12 ± 0.07	<0.001
Pat5	60.0 ± 0.0	0.46 ± 0.00	0.062	60.0 ± 0.0	0.46 ± 0.00	0.062
Pat9	50.0 ± 0.0	0.9 ± 0.123	0.476	50.0 ± 0.0	0.90 ± 0.08	0.459
Pat10	33.3 ± 0.0	1.08 ± 0.09	0.783	33.3 ± 0.0	0.45 ± 0.05	0.348
Pat13	80.0 ± 0.0	0.18 ± 0.04	<0.001	90.0 ± 10.0	0.18 ± 0.05	<0.001
Pat14	80.0 ± 0.0	0.80 ± 0.00	0.043	80.0 ± 0.0	0.70 ± 0.10	0.029
Pat18	66.7 ± 0.0	0.20 ± 0.02	0.001	83.3 ± 0.0	0.15 ± 0.02	<0.001
Pat20	80.0 ± 0.0	0.15 ± 0.00	<0.001	100.0 ± 0.0	0.15 ± 0.00	<0.001
Pat21	75.0 ± 0.0	0.43 ± 0.00	0.025	100.0 ± 0.0	0.41 ± 0.02	0.001
Pat23	80.0 ± 0.0	1.67 ± 0.00	0.281	100.0 ± 0.0	0.83 ± 0.17	0.005
Ave	67.9 ± 0.8	0.60 ± 0.01	n.a	78.5 ± 0.9	0.44 ± 0.04	n.a

**Table 5:** The performance of CSSPM with and without Gaussian augmentation (average of all 11 patients).

Whether to adopt Gaussian augmentation	Sensitivity (%)	FPR (h)
CSSPM (without augmentation)	75.4 ± 0.7	0.49 ± 0.03
CSSPM (with augmentation)	**78.5** ± **0.9**	**0.44** ± **0.04**

## Data Availability

The CHB-MIT Scalp EEG Dataset is openly available in PhysioNet via https://doi.org/10.13026/C2K01R.
